# ErbB2 and p38γ MAPK mediate alcohol-induced increase in breast cancer stem cells and metastasis

**DOI:** 10.1186/s12943-016-0532-4

**Published:** 2016-07-14

**Authors:** Mei Xu, Zhenhua Ren, Xin Wang, Ashley Comer, Jacqueline A. Frank, Zun-ji Ke, Yi Huang, Zhuo Zhang, Xianglin Shi, Siying Wang, Jia Luo

**Affiliations:** Department of Pharmacology and Nutritional Sciences, University of Kentucky College of Medicine, Lexington, KY 40536 USA; Pathophysiological Department, School of Basic Medicine, Anhui Medical University, Hefei, Anhui 230032 China; Department of Biochemistry, Shanghai University of Traditional Chinese Medicine, Shanghai, 201203 China; Department of Surgery, North Shore Long Island Jewish Health System-Hofstra University School of Medicine, Manhasset, NY USA; Department of Toxicology and Cancer Biology, University of Kentucky College of Medicine, Lexington, KY 40536 USA

**Keywords:** Alcohol, Cancer stem cell, p38 gamma, MCF7-ErbB2, Metastasis, Tumor promotion

## Abstract

**Background:**

Both epidemiological and experimental studies suggest that excessive alcohol exposure increases the risk for breast cancer and enhances metastasis/recurrence. We have previously demonstrated that alcohol enhanced the migration/invasion of breast cancer cells and cancer cells overexpressing ErbB2/HER2 were more sensitive to alcohol exposure. However, the underlying mechanisms remain unclear. This study was designed to investigate the mechanisms underlying alcohol-enhanced aggressiveness of breast cancer. Cancer stem cells (CSCs) play a critical role in cancer metastasis and recurrence.

**Methods:**

We evaluated the effect of chronic alcohol exposure on mammary tumor development/metastasis in MMTV-neu transgenic mice and investigated the cell signaling in response to alcohol exposure in breast cancer cells overexpressing ErbB2/HER2.

**Results and discussion:**

Chronic alcohol exposure increased breast cancer stem cell-like CSC population and enhanced the lung and colon metastasis in MMTV-neu transgenic mice. Alcohol exposure caused a drastic increase in CSC population and mammosphere formation in breast cancer cells overexpressing ErbB2/HER2. Alcohol exposure stimulated the phosphorylation of p38γ MAPK (p-p38γ) which was co-localized with phosphorylated ErbB2 and CSCs in the mammary tumor tissues. In vitro results confirmed that alcohol activated ErbB2/HER2 and selectively increased p-p38γ MAPK as well as the interaction between p38γ MAPK and its substrate, SAP97. However, alcohol did not affect the expression/phosphorylation of p38α/β MAPKs. In breast cancer cell lines, high expression of ErbB2 and p-p38γ MAPK was generally correlated with more CSC population. Blocking ErbB2 signaling abolished heregulin β1- and alcohol-stimulated p-p38γ MAPK and its association with SAP97. More importantly, p38γ MAPK siRNA significantly inhibited an alcohol-induced increase in CSC population, mammosphere formation and migration/invasion of breast cancer cells overexpressing ErbB2.

**Conclusions:**

p38γ MAPK is downstream of ErbB2 and plays an important role in alcohol-enhanced aggressiveness of breast cancer. Therefore, in addition to ErbB2/HER2, p38γ MAPK may be a potential target for the treatment of alcohol-enhanced cancer aggressiveness.

**Electronic supplementary material:**

The online version of this article (doi:10.1186/s12943-016-0532-4) contains supplementary material, which is available to authorized users.

## Background

Breast cancer is the most commonly diagnosed cancer and the second leading cause of cancer death among women in the United States [1]. Although the exact etiology for breast cancer is unclear, it is believed both genetics and environmental factors play an important role, and more likely it is the interplay of genetics and environmental factors that contribute to the carcinogenesis and progression of breast cancer. Alcohol abuse is one of the environmental factors that contribute to the etiology of breast cancer. Epidemiological studies indicate that alcohol consumption significantly increases the risk for breast cancer in a concentration- and duration-dependent manner [2–4]. In addition to the promotion of breast cancer carcinogenesis, alcohol may also enhance the growth of existing breast tumors and increases the aggressiveness of breast cancer cells to invade and metastasize [5–7]. The epidemiological findings are supported by experimental studies using various model systems which show that alcohol promotes mammary tumorigenesis/metastasis in animals, stimulates migration/invasion of breast tumor cells and enhances the expression of markers for epithelial-mesenchymal transition in cell culture systems [8–22]. However, the molecular mechanisms underlying alcohol promotion of breast cancer development and progression remain unclear.

Our previous studies have provided the evidence in which the interplay of alcohol exposure and genetic amplification caused enhanced aggressiveness of breast cancer cells. Overexpression of ErbB2 receptor is found in 20 ~ 30 % of breast cancer patients and is associated with poor prognosis and relapse [23, 24]. We showed that in culture systems breast cancer cells overexpressing ErbB2 were much more sensitive to alcohol-induced migration/invasion compared to those cells with low expression of ErbB2 [8, 12, 15]. However, several questions remain unanswered. For example, does an alcohol-induced increase in migration/invasion in ErbB2 overexpressing cells result in enhanced metastasis in animal models? What is the down-stream signaling of ErbB2 responsible for alcohol-enhanced aggressiveness of mammary tumors? Since, there is increasing evidence showing that cancer stem cells (CSC) play an important role in cancer aggressiveness [25–27], are CSCs involved in alcohol-induced tumor promotion? p38γ MAPK is one of four members of the p38 MAPK family [28]. Recent studies indicate that p38γ MAPK is implicated in breast cancer progression and aggressiveness [29]. We hypothesize that alcohol may enhance the aggressiveness of breast cancer cells by stimulating the ErbB2/p38γ MAPK pathway and activating CSCs. With both in vitro and in vivo approaches, we show that alcohol increases CSC population in ErbB2 overexpressing breast cancer cells; alcohol enhances the lung and colon metastasis and CSC population in MMTV-neu transgenic mice. p38γ MAPK is downstream of ErbB2 and ErbB2/p38γ signaling pathway and it plays an important role in alcohol-induced aggressiveness of breast cancer cells.

## Methods

### Materials

ALDEFLUOR kits and MammoCult™ Human Medium Kit were purchased from Stemcell Technologies (Vancouver, Canada). Ultra low cluster plates were obtained from Corning Incorporated (Corning, NY). Anti-phospho-Her2/ErbB2 (Tyr1248) and ErbB2 polyclonal antibodies were purchased from Cell Signaling Technology Inc. (Beverly, MA). Polyclonal anti-phospho-p38 gamma (p-p38γ) (Thr180/Tyr182) antibody was produced by us in collaboration with 21st Century Biochemicals (Marlboro, MA). FITC conjugated anti-mouse/human CD44 and PE conjugated CD24 antibodies were purchased from BioLegend (San Diego, CA). Protein A/G beads were obtained from Santa Cruz Biotechnology (San Diego, CA). Polyclonal anti-phospho-p38 MAPK (Thr180/Tyr182) antibody and anti-phospho-Her2/ErbB2 (Tyr1248) (monoclonal) were purchased from Life Technologies (Carlsbad, CA) and Cell Signaling Technology Inc. (Beverly, MA), respectively. Anti-Neu/Her2/ErbB2 (monoclonal), p38α, p38γ and SAP97 antibodies were purchased from Santa Cruz Biotechnology (San Diego, CA). Anti-GAPDH antibody was obtained from Research Diagnostics, Inc. (Concord, MA). Anti-phosphoserine/threonine antibody was obtained from Abcam Inc. (Cambridge, MA). p38γ shRNA and control shRNA were purchased from Santa Cruz Biotechnology (San Diego, CA). Matrigel Invasion Chambers were purchased from BD Biosciences (Bedford, MA). Transwell was obtained from Costar Corp. (Acton, MA). Antibiotic-Antimycotic (Anti-Anti) and cell culture mediums were obtained from Gibco (Life Technologies). All other chemicals were obtained from Sigma-Aldrich (St. Louis, MO).

### Cell culture and alcohol exposure method

MCF7 cells were grown in DMEM medium containing 10 % fetal bovine serum (FBS) and 1 % Antibiotic-Antimycotic (Additional file 1: Figure S1) . MCF7-ErbB2 cells were cultured in full DMEM medium with hydrocortisone (1 μg/ml) and insulin (10 μg/ml). Hs578T cells were cultured in full DMEM medium with insulin. BT474 cells were cultured in full RPMI medium with insulin. SKBR3 cells were cultured in full IMEM medium. Physiologically relevant concentrations of alcohol (100, or 200 mg/dl) were used in this study [30]. A method utilizing sealed containers was employed to maintain alcohol concentrations in the culture medium. The containers were placed in a humidified environment and maintained at 37 °C with 5 % CO_2_. With this method, alcohol concentrations in the culture medium can be accurately maintained [31]. All cell lines were grown at 37 °C with 5 % CO_2_. For heregulin β1 or Tyrphostin AG 825 (AG825) treatment, cells were serum starved overnight, pretreated with or without DMSO or AG825 (10 or 50 μM) for 2 h, followed by heregulin β1 (50 ng/ml) or alcohol exposure for the indicated times.

### Generation of phosphospecific antibody against p38γ MAPK

Affinity-purified antibodies specifically against the dual-phosphorylation motif, Thr-Gly-Tyr [32], located in the activation loop [Thr(p) 180/Tyr(p) 182] on p38γ MAPK were generated at 21st Century Biochemicals (Marlboro, MA). Rabbits were immunized with the phosphorylated p38γ peptide Acetyl-SEM[pT]G[pY]VVT-Ahx-C-amide and serum was affinity purified. Immuoprecipitation assay was applied to verify the specificity of the antibodies. We have verified that this antibody is specific for p- p38γ MAPK and does not cross-react with p38α/β MAPK (data not shown).

### Generation of cells stably expressing p38γ shRNA

Short hairpin RNA (shRNA) of p38γ (p38γsh) or scrambled control shRNA (consh) (Santa Cruz Biotechnology) was transfected into MCF7-ErbB2 or BT474 cells using a Neon Transfection machine (Life Technologies). Positive colonies were selected in standard cell culture media containing 4 μg/ml puromycin. Cell lysates were collected and analyzed by immunoblotting for the verification of the silencing of p38γ MAPK.

### ALDEFLUOR assay (Stem-like cell population assay)

The cancer stem-like cells (CSCs) were identified by measuring aldehyde dehydrogenase (ALDH) activity [26, 33]. The ALDEFLUOR assay (Stemcell Technologies) was performed according to the manufacturer’s protocol and the high ALDH enzymatic activity in cells were tested by using a flow cytometer as described previously [26, 33]. Briefly, after exposure to alcohol (0, 100 or 200 mg/dl) for the indicated time, 10^6^ cells were incubated in ALDEFLUOR assay buffer containing ALDH substrate (1 μmol/l per 1 × 10^6^ cells) for 40 min at 37 °C. Meanwhile, an aliquot of cells was treated under identical conditions with a specific ALDH inhibitor [50 mmol/l, diethylaminobenzaldehyde (DEAB)] as a negative control. CSCs were identified using a FACSCalibur (Becton Dickinson) flow cytometer and analyzed using the WINMDI software. The results were expressed relative to control groups.

### Flow cytometry (CD24/CD44 Assay)

The expression of cell surface markers (CD44 and CD24) on MCF7 or MCF7-ErbB2 cells was analyzed by flow cytometric assay. Briefly, cells with or without ethanol treatments were suspended in PBS containing 2 % BSA (10^6^ cells/100 ul). Combinations of FITC-CD44 and PE-CD24 or their respective isotype controls were added to the cell suspension at the concentrations recommended by the manufacturer, and then incubated at 4 °C in the dark for 30 min. The labeled cells were washed with PBS and then analyzed on a FACSCalibur (Becton Dickinson) flow cytometer and the WINMDI software.

### Assaying mammosphere formation

Mammosphere culture was performed as described previously [34, 35]. Briefly, after alcohol treatment, cells were plated as single cell suspension in ultra-low attachment 24-well plates (Corning) at 1000 cells/well. Cells were grown in serum-free MammoCult™ Human Medium (Stemcell Technologies) for 10 days. The images of mammospheres were captured using a Zeiss Axiovert 40C photomicroscope. The number of mammospheres in each well that were 60 μm or larger in size were counted according to the manufacturer’s protocol (MammoCult™ Human Medium, Stemcell Technologies) and expressed relative to control groups.

### Immunoblotting and immunoprecipitation

Cells or frozen tumor tissues were lysed in modified RIPA buffer (150 mM NaCl, 50 mM Tris, 1 % NP-40, 0.25 % sodium deoxycholate) containing 1 mM sodium vanadate, 1 mM phenylmethanesulfonyl fluoride (PMSF), 5 μg/ml of aprotinin, and 2 μg/ml of leupeptin. The procedure for immunoblotting has been previously described [22]. Briefly, protein samples were clarified by centrifugation at 14,000 rpm for 10 min at 4 °C and were resolved by sodium dodecyl sulfate-polyacrylamide gel electrophoresis (SDS-PAGE). The separated proteins were transferred to nitrocellulose membranes. The membranes were probed with indicated primary antibodies, followed by the appropriate horseradish peroxidase-conjugated secondary antibodies, and developed by enhanced chemiluminescence. The intensity of specific proteins was quantified using Carestream Molecular Image Software.

For immunoprecipitation, equal amount of proteins (about 500–800 μg) were incubated with anti-p38γ, p38α/β or SAP97 antibodies, respectively, overnight at 4 °C, followed by treatment with Protein A/G beads conjugated to agarose for 4 h at 4 °C. Immunoprecipitates were collected by centrifugation at 5,000 g for 5 min at 4 °C. Samples were washed 5X with RIPA buffer, 1X with cold-TBS, and boiled in sample buffer (187.5 mM Tri-HCl, pH 6.8, 6 % SDS, 30 % glycerol, 150 mM DTT and 0.03 % bromophenol blue). Proteins were resolved in SDS-PAGE and analyzed by immunoblotting.

### Assaying cell migration and invasion

Cell migration was analyzed using a Transwell Migration System (Costar). Cell invasion was assayed using Matrigel Invasion Chambers (BD Biosciences). Briefly, after alcohol exposure for 10 days, equal amount of cells were placed on the upper compartment of the Transwell chambers or invasion chambers in serum free medium. Culture medium containing 10 % FBS was added into the lower compartment of invasion/migration chambers and served as chemoattractants for the cells. The chambers were cultured at 37 °C in 5 % CO_2_ in the presence/absence of alcohol (100 mg/dl) for 12 h. Cells were fixed in 4 % paraformaldehyde and stained with 0.5 % crystal violet in 2 % ethanol. Membranes were washed and the cells that remained on the top of the invasion/transwell inserts were removed (non-migrated cells). The dye was eluted with 10 % acetic acid and the absorbance was measured at 595 nm using a microtiter platereader (Beckman coulter).

### Alcohol exposure in MMTV-neu transgenic mice

FVB MMTV-neu transgenic mice were obtained from Jackson Laboratory (Bar Harbor, MA). All procedures were performed in accordance with the guidelines set by the National Institutes of Health (NIH) Guide for the Care and Use of Laboratory Animals and were approved by the Institutional Animal Care and Use Committee. FVB MMTV-neu transgenic mice develop spontaneous mammary tumors in 8–10 months (5). Mice (12 weeks old without tumors) were separated into two groups. For the alcohol-exposed group (*n* = 11), mice were fed with an alcohol liquid diet (Bio-Serv, Flemington, NJ) containing 6.7 % v/v ethanol. Mice in the control groups (*n* = 12) received the liquid diet without ethanol but with equal caloric supplementation. Tumorigenesis and size of tumor was monitored weekly. Mice with tumors exceeding 20 mm maximum diameter were euthanized and metastasis was analyzed as previously described [18]. Blood was collected in the early morning from the mouse tails and alcohol concentration was analyzed by Alcohol Analyser AM1 (Analox Instruments, MA). Mammary tumor tissues were fixed and processed for immunostaining or frozen in −80 °C for immunoblotting analysis.

### Immunofluorescent staining

Immunofluorescent (IF) staining was performed as described [36]. Briefly, tumor tissues were removed and fixed with 4 % paraformaldehyde and then transferred to 30 % sucrose. Tissues were sectioned at 5 μm thickness with a Cryostat Microtone (Thermo Scientific). Tissue sections were rinsed in PBS, blocked by 1 % BSA for 1 h, and then incubated with indicated primary antibodies (1:300) (FITC-CD44, p-p38γ, pErbB2) overnight at 4 °C. After washing with PBS, sections were incubated with appropriate fluorescent conjugated secondary antibodies for 1 h at room temperature. Images were photographed using an inverted Olympus 1X81 microscope. The fluorescent intensity was analyzed by ImageJ software and calculated relative to the control groups.

### Statistics

Differences among treatment groups were analyzed using analysis of variance (ANOVA). Differences in which *p* was less than 0.05 were considered statistically significant. In cases where significant differences were detected, specific *post-hoc* comparisons between treatment groups were examined with Student-Newman-Keuls tests. The prevalence of metastasis between control and ethanol-treated groups was determined by the Fisher exact test.

## Results

### Alcohol increases cancer stem like cell (CSC) population in breast cancer cells overexpressing ErbB2

We previously demonstrated that breast cancer cells overexpressing ErbB2 are much more sensitive to alcohol-induced migration/invasion compared to those cells with a low level of ErbB2 [8, 12, 15]. In this study, we sought to determine whether alcohol affects CSC and the potential role of ErbB2 in the regulation of CSC. We first examined the effect of alcohol on MCF7 breast cancer cells and MCF7 cells overexpressing ErbB2 (MCF7-ErbB2). MCF7 or MCF7-ErbB2 cells were treated with alcohol (0, 100 or 200 mg/dl) for 10 or 20 days, and CSC population was determined by aldehyde dehydrogenase (ALDH) activity which was measured with an ALDEFLUOR assay. This assay has been successfully used to determine CSC population in breast cancer cells [26, 33]. In non-alcohol-treated control cells, MCF7-ErbB2 cells had more basal CSC population than MCF7 cells (Fig. 1a and Additional file 2: Figure S2). Alcohol exposure significantly increased CSC population in both MCF7 and MCF7-ErbB2 cells; however, alcohol-induced increase of CSC in MCF7-ErbB2 cells was much more than that of MCF7 cells. Alcohol increased CSC population in MCF7-ErbB2 cells in a concentration and duration-dependent manner (Fig. 1b). However, short term exposure to alcohol (12 ~ 48 h) did not significantly alter CSC population (data not shown). One of the characteristics for mammary CSCs is to form mammospheres in an ultra-low attaching culture condition. As shown in Fig. 1c and d, alcohol significantly increased mammosphere formation in both MCF7-ErbB2 cells and BT474 cells; BT474 cells are another breast cancer cell line with a high expression of ErbB2. However, alcohol did not affect mammosphere formation in MCF7 cells.

**Fig. 1:** Effect of alcohol on cancer stem-like cell (CSC) population. **a** MCF7 or MCF7-ErbB2 cells were exposed to alcohol (0 or 100 mg/dl) for 10 days, and then were processed for ALDEFLUOR assay, followed by flow cytometry for the detection of CSCs as described in the Materials and Methods. CSC population was calculated as percentage of total cells population. Each data point was mean ± SEM of three independent experiments. *denotes significant difference from respective control groups. #denotes significant difference from alcohol-treated MCF7 cells. **b** MCF-ErbB2 cells were exposed to alcohol (0, 100 or 200 mg/dl) for 10 or 20 days and then CSC population was determined as described above. *denotes significant difference from respective control groups. #denotes significant difference from respective 10 day-alcohol-exposed groups. δ denotes significant difference from 100 mg/dl alcohol-exposed groups during the 20 day exposure period. **c** and **d** MCF7, MCF7-ErbB2 or BT474 cells were exposed to alcohol (0 or 100 mg/dl) for 10 days, then 1000 cells were cultured on ultra-low attachment plates for assaying mammosphere formation as described in the Materials and Methods. The cell morphology was captured by a Zeiss Axiovert 40C photomicroscope. The number of mammospheres was determined. Each data point was the mean ± SEM of three independent experiments. *denotes significant difference from respective control groups. #denotes significant difference from alcohol-treated MCF7 cells. Bar = 50 μm. **e** and **f** Expression of breast cancer stem cell markers CD44^+^/CD24^−^ in MCF7 (**e**) or MCF7-ErbB2 (**f**) cells treated with or without Ethanol (100 mg/dl) was determined by flow cytometry. All experiments were repeated at least three times and there were triplicates for each replication. Each data point was the mean ± SD of three independent experiments

The alcohol-increased CSCs in MCF7 and MCF7-ErbB2 cells were confirmed by measuring the cell surface markers of CD44^+^/CD24^-/low^. The expression of CD44^+^/CD24^-/low^ has been extensively used as markers for breast cancer stem cells. We examined the expression of CD44^+^/CD24^-/low^ in MCF7 and MCF7-ErbB2 cells by flow cytometric assay (Fig. 1e and f). The results revealed much more CD44^+^/CD24^-/low^ positive cells, indicating a high ratio of cancer stem cells in MCF7-ErbB2 cell which was also observed in the ALDH assay. We also compared the ratio of CD44^+^/CD24^-/low^ cells in MCF7 and MCF7-ErbB2 treated with or without ethanol. Ethanol exposure enhanced the expression of CD44^+^/CD24^-/low^ in both cells, but to a greater extent in MCF7-ErbB2 cells (Fig. 1f).

### Alcohol exposure enhances metastasis and increases CSC in MMTV Neu transgenic mice

FVB MMTV Neu transgenic mice expressing high levels of neu (ErbB2 in human) develop spontaneous mammary tumors in about 8–10 months (5). These mice were exposed to alcohol by feeding with a liquid diet containing 0 or 6.7 % ethanol. This paradigm of alcohol exposure resulted in a blood alcohol concentration (BAC) of nearly 100 mg/dl which is equivalent to the level of human intoxication (Fig. 2a). We measured the metastasis when the maximum diameter of the tumor reached 20 mm. The percentage of mice showing lung metastasis in control and alcohol-fed mice was 16.7 and 81.8 %, respectively; while colon metastasis was 0 and 45.4 %, respectively (Fig. 2b). Recent evidence indicates that CSC population is a driving force for cancer malignance/metastasis. We therefore examined the effect of alcohol on CSCs in MMTV Neu transgenic mice. Breast CSCs are characterized as the CD44+/CD24- population [15, 17, 18]. We showed that alcohol exposure increased CD44+ cells, implying an increase in CSCs (Fig. 2c and d).

**Fig. 2:** Effect of alcohol on cancer metastasis in FVB MMTV Neu mice. **a** FVB MMTV Neu mice were fed with liquid diet containing ethanol (0 or 6.7 %) for about 12 months, blood alcohol concentration (BAC) was measured as described in Materials and Methods. **b** After the maximal diameter of tumors reached 20 mm_,_ mice were sacrificed and analyzed for tumor metastasis as described in the Material and Methods. **c** and **e** The mammary tumor tissues were fixed, sectioned, and processed for immunofluorescent staining with indicated antibodies as described in the Material and Methods. Bar = 40 μm (**c**), 25 μm (**e**). **d** and **f** The intensity of CD44 (**d**), p-p38γ, CD44 or pErbB2 (**f**) in (**c**) and (**e**) were measured using ImageJ. The relative levels were quantified and normalized to the controls. **g** and **h** The mammary tumor tissues were collected and the expression of phosphorylated ErbB2 (pErbB2) and p38γ MAPK (p-p38γ) was determined by immunoblotting (*N* = 4). The relative levels of pErbB2 and p-p38γ were quantified and normalized to the loading control (Ponceau S stain). Each data point was the mean ± SEM of three independent experiments. *denotes significant difference from control groups (*p* < 0.05)

### Alcohol activates ErbB2/p38γ MAPK signaling pathway

We next determined whether alcohol activated ErbB2 in MMTV Neu mice and what were the downstream signals of ErbB2. p38γ MAPK has been implicated in the aggressiveness of breast cancer cells [29]. Alcohol increased the phosphorylation of ErbB2 and p38γ MAPK which was revealed by the immunofluorescent staining of fixed tumor tissues (Fig. 2e and f). Alcohol-induced pErbB2 and p-p38γ were co-localized in CD44+ cells, suggesting that ErbB2/p38γ signaling was involved in alcohol promotion of CSCs. This was confirmed by immunoblotting analysis on mammary tissue samples (Fig. 2g and h). It appeared that alcohol treatment also increased the expression of ErbB2. To further evaluate the effect of alcohol on ErbB2/p38γ MAPK signaling pathway, we treated MCF7-ErbB2 cells with alcohol (0, 100 or 200 mg/dl) for 10 days, and then examined the phosphorylation of ErbB2 (Tyr1248) and p38γ MAPK (Thr180/Tyr182). Alcohol activated ErbB2 and p38γ MAPK in MCF7-ErbB2 cells (Fig. 3a), but not other isoforms of p38 MAPK (Fig. 3b). The synapse-associated protein (SAP97), also known as disks large homolog 1 (DLG1) is a physiological substrate for the p38γ MAPK [37, 38]. We showed that alcohol promoted the interaction between p38γ MAPK and SAP97, and also increased the phosphorylation of SAP97 (Fig. 3c).

**Fig. 3:** Effect of alcohol on the activation of ErbB2 and p38γ MAPK. **a** MCF7-ErbB2 cells were exposed to alcohol (0, 100 or 200 mg/dl) for 10 days, then cell lysates were collected and the expression of phosphorylated ErbB2 and p38γ MAPK (pErbB2 and p-p38γ) was analyzed by immunoblotting. GAPDH served as loading controls. **b** Equal amount of proteins were immunoprecipitated (IP) with an anti-p38α/β antibody, then immunoblotted (IB) using an anti-pan-phosphorylated p38 MAPK antibody (p-p38). **c** MCF7-ErbB2 cells stably expressing control shRNA or shRNA for p38γ MAPK were exposed to alcohol (0 or 100 mg/dl) for 10 days, then cells lysates were collected. Equal amount of proteins were immunoprecipitated (IP) with an anti-SAP97 antibody, then immoblotted (IB) with antibodies directed against phosphorylated serine/threonine antibody and p38γ MAPK. The experiment was replicated three times

### The expression ErbB2 and p38γ MAPK is positively correlated to CSC population in breast cancer cell lines

We showed that alcohol increased CSC population and activated ErbB2/p38γ MAPK pathway. We sought to determine whether more CSC population correlated to a high activity of ErbB2/p38γ MAPK in breast cancer cell lines. As shown in Fig. 4a and b, MCF7-ErbB2 cells expressed more p38γ MAPK, particularly phosphorylated p38γ MAPK and had significantly more CSC population compared to MCF7 cells. We further compared six other breast cancer cell lines for the expression of ErbB2/p38γ MAPK and CSC population (Fig. 4c and d). Generally, high expression of ErbB2 and phosphorylated p38γ MAPK was correlated with more CSC population.

**Fig. 4:** Correlation of the expression of ErbB2, p38γ MAPK, p-p38γ and CSC population (ALDEFLUOR positive cells). **a** The expression of ErbB2, p38γ, p-p38γ and p38α in MCF7 and MCF7-ErbB2 cells was analyzed by immunoblotting. **b** CSC population in these cells was measured by ALDEFLUOR assay followed by flow cytometry. **c** The expression of ErbB2, p38γ, p-p38γ and p38α in various breast cancer cells was analyzed by immunoblotting. **d** CSC population in these cells was determined as described above. The experiment was replicated three times

### p38γ MAPK is down-stream of ErbB2

The relationship between ErbB2 and p38γ has never been explored. To better understand ErbB2/p38γ MAPK signaling pathway, we treated MCF7-ErbB2 cells with heregulin β1 to activate ErbB2, and then determine the phosphorylation of p38γ MAPK. MCF7-ErbB2 cells were treated with heregulin β1 (50 ng/ml) for the indicated time (0–6 h). Using commercial antibodies for p38γ MAPK and phosphorylated p38 MAPK, we showed that heregulin β1 increased the phosphorylation of p38γ MAPK in MCF7-ErbB2 cells by immunoprecipitation assay (Fig. 5a). It appeared that the peak activation for ErbB2 and p38γ was around 30 min and 60 min after heregulin β1 treatment, respectively. Similar results were observed in BT474 cells, a breast cancer cell line naturally expressing high levels of ErbB2 (Fig. 5b). But in BT474 cells, the peak activation for ErbB2 was around 60 min and lasted longer while the peak activation for p38γ was around 180 min following heregulin β1 treatment. We have generated a phospho-specific antibody directed against p38γ MAPK in collaboration with 21st Century Biochemical (Marlboro, MA). The results from this antibody were consistent with the data presented in Fig. 5a, confirming that heregulin β1 activated p38γ MAPK in MCF7-ErbB2 cells (Fig. 5c). Heregulin β1 also increased the interaction of p38γ MAPK with its substrate, SAP97, as well as the phosphorylation of SAP97 (Fig. 5d). The inhibition of ErbB2 activation by the pretreatment of Tyrphostin AG 825 (AG825) blocked heregulin-induced phosphorylation of ErbB2 and p38γ MAPK (Fig. 5e and g). In addition, AG825 attenuated heregulin β1-increased p38γ-SAP97 interaction (Fig. 5f and h). Together, these results suggested that activation of ErbB2 induced the phosphorylation of p38γ MAPK and promoted its interaction with its substrates.

**Fig. 5:** Effect of heregulin β1 on the activation of ErbB2, p38γ MAPK and SAP97. **a** MCF7-ErbB2 cells were treated with heregulin β1 (50 ng/ml) for the indicated times. The phosphorylation of ErbB2 (pErbB2) was determined by immunoblotting. The phosphorylation of p38γ was analyzed by immunoprecipitation. Cell lysates were first immunoprecipitated (IP) by an anti-p38γ antibody and then immunoblotted (IB) with an anti-pan-phosphorylated p38 MAPK. The experiment was replicated three times. **b** The heregulin β1-induced phosphorylation of ErbB2 and p38γ in BT474 cells was determined. The notations are the same as in panel (**a**). **c** The heregulin β1-induced phosphorylation of p38γ MAPK in MCF-ErbB2 cells was determined by immuoblotting using a phospho-specific antibody directed against p38γ MAPK (p-p38γ). **d** MCF7-ErbB2 cells were treated with heregulin β1 for indicated times. Equal amount of proteins were immunoprecipitated (IP) with an anti-SAP97 antibody, then immunoblotted (IB) using antibodies directed against phosphorylated serine/threonine or p38γ MAPK. **e** MCF7-ErbB2 cells were pretreated with DMSO or AG825 (50 μM) for 2 h followed by heregulin β1 treatment. The phosphorylation of ErbB2 and p38γ MAPK was determined by immunoblotting. **f** MCF7-ErbB2 cells were pretreated with DMSO or AG825 (50 μM) for 2 h followed by heregulin β1 treatment. The interaction of p38γ MAPK and SAP97 was determined by immunoprecipitation. Equal amount of protein were immunoprecipitated (IP) with an anti-p38γ antibody, then immnoblotted (IB) with an anti-SAP97 or anti-p38γ MAPK antibody. The experiment was replicated three times. **g** and **h** The relative levels of p-p38γ and SAP97 were quantified, normalized to the loading control, and then expressed relative to time 0 in either DMSO or AG825 groups. Each data point was the mean ± SEM of three independent experiments. *denotes significant difference from control groups (*p* < 0.05)

### Inhibition of ErbB2 blocks alcohol-activated p38γ MAPK

To determine whether ErbB2 played a role in alcohol-induced activation of p38γ MAPK, MCF7-ErbB2 cells were exposed to alcohol (10–360 min). Meanwhile, we blocked ErbB2 activation by pretreating MCF7-ErbB2 cells with AG825. As shown in Fig. 6a, AG825 blocked alcohol-induced phosphorylation of ErbB2 and p38γ MAPK. However, acute alcohol exposure (10–360 min) did not affect SAP97 phosphorylation (Fig. 6b). Although acute alcohol exposure activated p38α/β (Fig. 6c), AG825 failed to block alcohol-induced activation of p38α/β (Fig. 6c).

**Fig. 6:** Effect of ErbB2 inhibitor on alcohol-induced activation of ErbB2, p38γ MAPK and SAP97. **a** MCF7-ErbB2 cells were pretreated with DMSO or AG825 (10 μM) for 2 h, followed by alcohol exposure (0 or 200 mg/dl) for indicated times. The phosphorylation of ErbB2 or p38γ was determined by immunoblotting. **b** The effect of alcohol on the phosphorylation of SAP97 at serine/threonine sites was determined by immunoprecipitation. Cell lysates were IP with an anti-SAP97 antibody and then IB with an antibody directed against phosphorylated serine/threonine. **c** MCF7-ErbB2 cells were pretreated with DMSO or AG825 (10 μM) for 2 h, followed by alcohol exposure (0 or 200 mg/dl) for indicated times. Equal amount of protein were IP with an anti-p38α/β antibody, then IB with an anti-pan-phosphorylated p38 MAPK antibody. The experiment was replicated three times

### p38γ MAPK mediates alcohol-increased mammosphere formation, CSC population and the migration/invasion of breast cancer cells

To confirm the involvement of p38γ MAPK in alcohol-enhanced CSCs and aggressiveness, we knocked down the expression of p38γ MAPK in MCF7-ErbB2 and BT474 cells by stably expressing either the control shRNA (Consh) or shRNA for p38γ MAPK (p38γsh) (Fig. 7a and b); p38γsh decreased the expression of p38γ MAPK by approximately 60 %. Knocking down p38γ MAPK abolished alcohol-induced interaction between p38γ MAPK and SAP97 (Fig. 3c). As shown in Fig. 7c and d, Knocking down p38γ MAPK blocked alcohol-induced formation of mammospheres in both MCF7-ErbB2 and BT474 cells. Knocking down p38γ MAPK also inhibited alcohol-increased CSC population (Fig. 7e). It was interesting to note that knocking down p38γ MAPK decreased basal mammospheres and CSC population, supporting its role in these processes. Furthermore, Knocking down p38γ blocked alcohol-stimulated migration and invasion in MCF7-ErbB2 cells (Fig. 7f and g). These results suggested that p38γ MAPK played an important role in alcohol-promoted aggressiveness of breast cancer cells.

**Fig. 7:** Effect of knocking down p38γ MAPK on alcohol-induced tumor promotion. **a** The expression of p38γ and p38α MAPK in MCF7-ErbB2 cells stably expressing control shRNA (Consh) or p38γ shRNA (p38γsh) was determined by immunoblotting. **b** The relative levels of p38γ in Consh and p38γsh-treated cells were quantified and expressed relative to Consh-treated group. **c** and **d** MCF7-ErbB2 and BT474 cells stably expressing control Consh or p38γsh were exposed to alcohol (0 or 100 mg/dl) for 10 days. After alcohol exposure, 1000 cells/well were cultured on ultra-low attachment plates for 10 days. The number of mammospheres was counted and calculated relative to the control groups treated with Consh. **e** After alcohol exposure for 10 days, the CSC population (ALDEFLUOR positive cells) in MCF7-ErbB2 cells stably expressing control shRNA (Consh) and p38γ shRNA (p38γsh) was determined by ALDEFLUOR assay followed by flow cytometry as described in the Materials and Methods. **f** and **g** After alcohol exposure for 10 days, MCF7-ErbB2 cells stably expressing control shRNA (Consh) or p38γ shRNA (p38γsh) were assayed for migration and invasion as described in the Materials and Methods. Each data point was the mean ± SEM of three independent experiments and expressed relative to control groups. *denotes significant difference between non-alcohol-treated groups (p38γsh-treated controls vs Consh-treated controls). #denotes significant difference from respective alcohol-exposed cells expressing p38γsh

## Discussion

We show here that alcohol exposure enhances the aggressiveness of breast cancer cells overexpressing ErbB2, which is evident by a significant increase in CSC population, mammosphere formation, migration/invasion as well as metastasis in MMTV-neu transgenic mice. Alcohol selectively stimulates the phosphorylation of p38γ MAPK (p-p38γ) which is down-stream of ErbB2. More importantly, down-regulation of p38γ MAPK by shRNA significantly inhibits alcohol-induced increases in CSC population, mammosphere formation and migration/invasion of breast cancer cells overexpressing ErbB2.

We have previously demonstrated that alcohol stimulated the migration/invasion in breast cancer cells over-expressing ErbB2 [21, 22]. The current study not only furthers the study by showing alcohol increasing CSC population and mammosphere formation, but confirms it in a more relevant mouse model, MMTV-neu transgenic mice. There are a number of techniques/assays for the characterization of CSCs. So far, a striking feature is that there is relatively little overlap between the different CSC markers reported in different tumor types or species [39]. ALDEFLUOR assay is based on the ALDH activity, while CD24 low/CD44+ assay is based on the expression of CD24/CD44 on cell surface. Both assays are extensively used to determine CSCs. Several studies compared these two assays and found that the overlap between ALDEFLUOR and CD24 low/Cd44+ assays was very low [33, 40]. In addition, one previous study showed that CD24 expression is reversely correlated with the ErbB2 expression which is consistent with our data [41]. The ratio of CSCs varies greatly among different cell types [26]. The current study focuses on alcohol-induced changes in breast CSCs. Our findings demonstrate that alcohol affects CSC in breast cancer cells overexpressing ErbB2 much more than cells with low ErbB2. Together, these results indicate that high expression of ErbB2 sensitizes breast cancer cells to alcohol exposure. A future study on human breast cancer patients is necessary to determine whether there is indeed an interaction among alcohol drinking, ErbB2 status and the aggressiveness/progression of breast cancer.

We have shown previously that alcohol induced the phosphorylation of ErbB2 in breast cancer cells over-expressing ErbB2 (21). However, the down-stream signaling components that mediate alcohol-enhanced aggressiveness remain unknown. The current study shows that alcohol selectively activates p38γ MAPK and blocking ErbB2 activation eliminates alcohol-induced phosphorylation of p38γ MAPK, indicating that p38γ MAPK is down-stream of ErbB2 signaling that is activated by alcohol exposure.

p38γ MAPK is relatively understudied compared to other isoforms in this family. p38γ MAPK is a member of the p38 MAPK family which has three other members, p38*α*, p38*β* and p38*δ*. These kinases share highly similar protein sequences; p38*α* and p38*β* are 75 % identical, whereas p38γ and p38*δ* are 62 and 61 % identical to p38*α*, respectively. In turn, p38γ and p38*δ* are *∼* 70 % identical to each other. The four p38 MAPK isoforms are widely expressed, although p38*β*, p38γ and p38*δ* expression appear to be higher in specific tissues; for example, p38*β* is abundant in brain, p38γ in skeletal muscle, and p38*δ* in endocrine glands [28]. In general, all p38 MAPKs are strongly activated by a wide variety of environmental and cellular stresses or by inflammatory cytokines and are poorly activated by serum or growth factors [28]. The canonical activation of p38 MAPKs occurs via dual phosphorylation of their Thr–Gly–Tyr motif, in the activation loop, by mitogen-activated protein kinase kinase (MKK) 3/6 (MKK3 and MKK6) [28]. Upon activation, the dually phosphorylated p38 MAPK goes through characteristic global conformational changes that alters the alignment of the two kinase halves (N-terminal and C-terminal domains) of the folded protein and enhances access to the substrate, which together increases enzymatic activity. To date, most studies of the p38 MAPK pathways focused on function of the p38α and p38*β* isoform, which is widely considered to negatively regulate malignant transformation; nonetheless, few reports address the p38γ and p38δ isoforms. Although p38γ and p38δ MAPK can phosphorylate typical p38 MAPK substrates such as the transcription factors ATF2, Elk-1 or SAP1, they cannot phosphorylate some substrates of p38*α* and p38*β* MAPK and have their unique substrates [28].

Recent studies indicate that p38γ MAPK may have some particular implications in breast cancer. For example, Meng et al. [42] showed that p38γ MAPK is overexpressed in highly metastatic human and mouse breast cancer cell lines and p38γ MAPK expression is preferentially associated with basal-like and metastatic phenotypes of breast tumor samples. Clinical evidence shows that elevated expression of p38γ MAPK is associated with lower overall survival of patients with breast cancer [29]. Using a computational mechanical model, Rosenthal et al. further showed that p38γ MAPK can regulate the changes of the cytoskeleton and cell shape of breast cancer cells and control cell motility. This evidence suggests an important role of p38γ MAPK in the aggressiveness of breast cancer. The current study for the first time establishes that p38γ MAPK may mediate alcohol-promoted aggressiveness of breast cancer cells.

Alcohol promotes the interaction between p38γ MAPK and its substrate, SAP97/DLG, causing SAP97/DLG phosphorylation (Fig. 3c). Heregulin β1 activates ErbB2/p38γ MAPK and also promotes p38γ MAPK/SAP97/DLG interaction (Fig. 5). These results indicate that alcohol activates the ErbB2/p38γ MAPK/SAP97/DLG pathway. SAP97/DLG is a scaffold protein and member of the membrane-associated guanylate kinase (PSD-MAGUK) family of multi-domain scaffolding proteins which recruits transmembrane and signaling molecules to localized plasma membrane sites [43]. SAP97/DLG has been known for its important role in neuron synapse assembly and plasticity [44]. SAP97/DLG is also present in epithelial cells and localized at the lateral membrane between cells [45]. It has been reported that SAP97/DLG is required for the polarization of migrating astrocytes [46]. A recent study showed that SAP97/DLG regulated the migration of non-small cell lung cancer cells [47]. However, the role of SAP97/DLG in the aggressiveness of breast cancer cells has not been established yet. A future study to investigate the involvement of SAP97/DLG in CSC and migration/invasion of breast cancer cells will provide insight into the *novel* function of SAP97/DLG in the context of cancer aggressiveness. It is interesting to note that unlike heregulin and long-term alcohol exposure, short-term alcohol exposure (up to 6 h) does not enhance p38γ MAPK/SAP97/DLG interaction. One possibility is that the effect of alcohol on ErbB2/p38γ MAPK/SAP97/DLG pathway is not strong enough that the changes in SAP97/DLG phosphorylation are beyond the detection of immunoblotting. Second possibility is that the time course of alcohol-induced p38γ MAPK/SAP97/DLG is different from that of heregulin and requires longer exposure to alcohol. Alcohol-induced activation of ErbB2/p38γ MAPK/SAP97/DLG pathway may be mediated through the production of reactive oxygen species (ROS). We have previously demonstrated that alcohol increases intracellular ROS accumulation in breast cancer cells and plays a role in alcohol-induced ErbB2 activation [15, 21]. In addition, the mitogen-activated protein kinase kinase 6 (MKK6), a major upstream kinase of p38γ MAPK and its activity is also regulated by intracellular ROS concentration [48].

## Conclusions

Breast cancer cells over-expressing ErbB2 are more sensitive to alcohol-promoted aggressiveness. Alcohol preferentially increases CSC population, mammosphere formation and migration/invasion in breast cancer cells overexpressing ErbB2. Chronic alcohol exposure enhances the lung and colon metastasis in MMTV-neu transgenic. Alcohol selectively activates p38γ MAPK which is down-stream of ErbB2. This study for the first time demonstrates ErbB2/p38γ MAPK/SAP97/DLG pathway may mediate alcohol-stimulated aggresiveness of breast cancer.

## Abbreviations

CSC, cancer stem-like cell; EtOH, ethanol; MAPK, mitogen-activated protein kinase; p38γ, p38 gamma; shRNA, short hairpin RNA

## Additional files

Additional file 1: Figure S1. Flow cytometry analysis of MCF7 cells cultured for 10 days in regular DMEM full medium or DMEM medium with hydrocortisone and insulin. After cultured in either regular DMEM full medium or DMEM medium with hydrocortisone and insulin for 10 days, MCF7 cells were processed for ALDEFLUOR assay **(A** and **B**) and CD24/CD44 assay (**C**). (EPS 1583 kb) Additional file 2: Figure S2. Flow cytometry analysis of MCF7 and MCF7-ErbB2 cells stained with ALDEFLUOR® (please see Materials and Methods). Gates (R1) were set according to DEAB control. **A**: MCF7 cells were treated with ethanol (0 or 100 mg/dl) for 10 days followed by ALDEFLUOR assay. **B**: MCF7-ErbB2 cells were treated with ethanol (0 or 100 mg/dl) for 10 days followed by ALDEFLUOR assay. All experiments were repeated at least three times and there were triplicates for each replication. (EPS 1244 kb)
